# Neuropsychological Impairment in Prodromal, First-Episode, and Chronic Psychosis: Assessing RBANS Performance

**DOI:** 10.1371/journal.pone.0125784

**Published:** 2015-05-14

**Authors:** TianHong Zhang, HuiJun Li, William S. Stone, Kristen A. Woodberry, Larry J. Seidman, YingYing Tang, Qian Guo, KaiMing Zhuo, ZhenYing Qian, HuiRu Cui, YiKang Zhu, LiJuan Jiang, Annabelle Chow, YunXiang Tang, ChunBo Li, KaiDa Jiang, ZhengHui Yi, ZePing Xiao, JiJun Wang

**Affiliations:** 1 Shanghai Mental Health Center, Shanghai Jiaotong University School of Medicine, Shanghai Key Laboratory of Psychotic Disorders, Shanghai 200030, PR China; 2 Florida A & M University, Department of Psychology, Tallahassee, Florida 32307, United States of America; 3 Harvard Medical School Department of Psychiatry, Beth Israel Deaconess Medical Center, 75 Fenwood Rd, Boston, MA 02115, United States of America; 4 Changi General Hospital, Department of psychological medicine, Singapore, Singapore; 5 Department of medical psychology, Faculty of Mental Health, Second Military Medical University, Shanghai 200433, China; Maastricht University, NETHERLANDS

## Abstract

**Background:**

Cognitive deficits are observed throughout all developmental phases of psychosis. However, prior studies have usually focused on a limited illness period and used a wide variety of cognitive instruments. Therefore, it has been difficult to characterize or highlight cognitive functioning in different stages of psychosis.

**Method:**

We administered the RBANS (Repeatable Battery for the Assessment of Neuropsychological Status) tests to 4 participant subgroups, including healthy volunteers (controls, HC, *n* = 28), subjects at high risk for clinical psychosis (prodrome, CHR, *n* = 27), first-episode schizophrenia patients (FE-Sz, *n* = 26), and mid-term and long-term chronic schizophrenia patients (Ch-Sz, *n* =147). Comparison, correlation, and regression analyses of RBANS index scores were assessed among groups. We examined clinical outcomes over 2 years between the CHR and HC subjects, and RBANS domains were used as possible predictors for conversion to psychosis.

**Results:**

Performance on all RBANS domains was significantly impaired during a post-onset stage of psychosis (FE-Sz and Ch-Sz), and RBANS scores declined along with disease progression. Regression analyses showed that for CHR and HC subjects, baseline impairment in delayed memory (DM) significantly predicted conversion to psychosis. Additionally, partial correlations showed that for FE-Sz and Ch-Sz subjects, DM was the only correlate with a later stage of psychosis.

**Conclusions:**

Cognitive deficits broadly emerged, and diminished functioning followed along with disease progression. Impairment in DM is perhaps one domain that helps us understand the development of psychosis. A critical need is to monitor and treat memory functioning for psychotic patients throughout all phases of the disease.

## Introduction

Cognitive deficits are a significant feature of psychosis, contributing to long-term disability and poor functional outcomes [1–3]. Underlying neurocognitive impairments at the post-onset phase of psychosis has received significant attention, with several studies reporting a number of cognitive domains, such as memory [4–6], attention [7, 8], language [9, 10] and visuospatial abilities [11, 12], being negatively impacted, especially during the late course of psychosis. Evidence points to the synchronization of neurobiological deteriorative processes that occurs along with the development of psychosis. Unfortunately however, such findings are fairly heterogeneous [13]. It is also imperative to identify and clearly distinguish the cognitive components that contributes to the progress of psychosis. This is because cognitive domains correspond to different functional brain regions and this has implications on our understanding of pathological mechanisms and neurobiology of psychosis.

Cognitive impairment has been observed in every stage of psychosis, even during the prodromal phase [14–16]. This suggests that cognitive dysfunction may not only be a consequence of chronic psychotic disorders, but it also precedes psychotic development and contributes to the onset of psychosis [17, 18]. Patterns of cognitive deficits can vary during the disease process. For instance, there might be an increase in the impairment of memory and attention rather than of language and visual functions in groups of schizophrenia (Sz) patients with clinical stability [19]. More severe deficits might be found in social cognition, language, and memory function among subjects with prodromal psychosis [14]. Although evidence from both cross-sectional and longitudinal studies are somewhat definitive, neuropsychological assessments are rather varied and multidimensional, which could be a barrier to fully understanding processes related to cognitive decline through the whole course of psychosis.

Few studies have covered the whole course of psychosis and have used relatively “standard” cognitive instruments. This makes it impossible to compare results on different stages of psychosis across studies. Meanwhile, both patients and clinicians desire a useful neuropsychological test battery for detecting the ongoing neurocognitive progression of psychosis. For psychotic patients, the test should be brief, not too time-consuming, and easily engaged. At the same time, Clinicians want a test with good reliability and validity, and which independently screens for positive symptoms of psychosis [19, 20]. Taking these two factors into account, the Repeatable Battery for the Assessment of Neuropsychological Status (RBANS) appears to be a viable option that has demonstrated these qualities for Chinese samples [21, 22].

Therefore the RBANS, a well-standardized cognitive battery, was used to examine neuropsychological changes over the development of psychosis. The current study profiled neuropsychological functioning among a wide range of psychotic patients in different stages of psychosis. Our hypothesis was that cognitive decline would occur across the whole course of psychosis, even at the pre-onset phase, and one or two subtypes of neuropsychological functional domains (such as attention or memory) might be more relevant/predictive of the development of psychosis. It was also expected that patients with a longer course of psychosis would show poorer neurocognitive performance.

## Method

### Sample

We enrolled 228 subjects who were assessed with the RBANS at a Shanghai-city-owned psychiatric hospital (Fig 1). Twenty-seven CHR subjects (clinical high risk, CHR group) and 26 first-episode schizophrenia (FE-Sz group) outpatients were consecutively drawn from Shanghai Mental Health Center (SMHC) between 2011 and 2013. The CHR group was recruited from an epidemiological survey conducted in 2011 [23], and detailed information regarding this survey has been published previously. A total of 89 participants identified with CHR by the SIPS/SOPS (Structured Interview for Prodromal Symptoms and the Scale of Prodromal Syndromes) [24, 25] in this epidemiological survey. Twenty-seven of the 89 CHR subjects volunteered to participate in the RBANS test at baseline. FE-Sz patients met DSM-IV diagnostic criteria for Sz through the SCID interview and had their first psychotic episode in the past year. These two groups met the following inclusion criteria: 1) age 15–45 years; 2) completed at least 6 years of education and able to understand the study; 3) their first visit to a mental health clinic for professional help; 4) no use of antipsychotic drugs at baseline; 5) having no documented organic or drug induced mental disorder, mental retardation, and severe somatic diseases (such as heart failure, cancer, etc.). Twenty-eight healthy controls (HC group) with a negative family history of mental disorders matched to the CHR group by age, gender, and education were recruited from the local community in Shanghai.

**Fig 1:** Sample flow diagram. The RBANS tests were administered to 228 subjects enrolled at SMHC between 2011 and 2013, including 28 HC, 27 CHR, 26 FE-Sz and 147 Ch-Sz.

One hundred and forty-seven patients with Sz were recruited from an inpatient unit at a psychiatric hospital. All patients were of the chronic type (chronic schizophrenia, Ch-Sz group), in stable condition, had been hospitalized for more than 2 years and mostly stayed at hospital. Those Ch-Sz patients had been receiving oral antipsychotic drugs with a stable dosage for at least 3 months. Physical examinations and laboratory tests were performed twice a year. None of the patients had a history of stroke, brain trauma, central nervous system infection, or seizure. All patients engaged in regular activities (such as watching TV, taking a walk in the hospital, playing cards, etc.) during their hospitalization. Patients were at times allowed to visit their guardians at home during weekends or holidays.

The Research Ethics Committee at the Shanghai Mental Health Center (SMHC) approved the study in 2011. All participants gave written informed consent. Those younger than 18 years of age in the CHR and FE-Sz group were signed up for the study by their parents, who provided consent. This Ch-Sz patient group was evaluated by nurses before signing in order to determine their ability to understand the consent form as well as the study.

### Instruments

#### CHR identification

The CHR status was determined based on the SIPS/SOPS interview. According to the SIPS/SOPS manual [24, 25], attenuated positive symptom syndrome (APSS) was defined as a rating of “3” and “5” for recent positive (P) symptoms (scales P1–P5) on the SOPS with sufficient frequency and duration. P symptoms referred to the existence of prodromal syndrome, including Unusual Thought Content, Suspiciousness, Grandiosity, Perceptual Abnormalities, and Disorganized Communication. Presence of Psychotic Symptoms (POPS) in the SIPS/SOPS was used to determine conversion into psychosis. This was defined by having P symptoms present at a psychotic level with a high intensity (Rated at level “6”) and at a sufficient frequency and duration/urgency.

The English version of the SIPS/SOPS has been widely used for identifying subjects with prodromal psychosis [26, 27] and has good inter-rater reliability and validity [25]. Our team members translated the SIPS/SOPS into Chinese and tested the Chinese version previously [28]. Details regarding the translated SIPS/SOPS can be found in our recent work [23]. We obtained good inter-rater reliability using the Chinese SIPS/SOPS (e.g., *r* = 0.96, *p* < 0.01 for the SOPS) and validity (26.4% of the sample transitioned into psychosis during the ensuing 2 years).

#### RBANS

The RBANS (Form A) [29] is a neuropsychological test battery that includes 12 subtests that form 5 age-adjusted index scores for the following cognitive abilities: Immediate Memory (IMM), Visuospatial/Constructional (VC), Language (LAN), Attention (ATT), and Delayed Memory (DEM), as well as a total cognitive functional score (TOT). The RBANS is suitable for comprehensive evaluation of neurocognitive functions among patients with Sz, and this test battery is suitable for use with Chinese samples [30–32]. Our research team previously assessed the reliability and validity of the Chinese version of the RBANS among a sample of schizophrenic patients [30]. This battery is a quality cognitive test for assessing patients with Sz [22].

### Procedures

All subjects received Form A of the RBANS test in a quiet room at baseline. Subjects in the CHR group were approached to take part in an epidemiological study [(detailed procedures are described elsewhere [23]] after completing the SIPS/SOPS interview. Subjects in the HC group were voluntary community members from Shanghai. A psychiatrist assessed the subject's current mental status and any family history of mental disorders using an unstructured interview. Subjects in the CHR or HC group were told they would be contacted in approximately 2 years to assess their mental health. Those subjects were followed up about 2 years later (at least twice in either March or April 2012 or November 2013), and conversion into psychosis was determined by POPS criteria. These subjects were then re-assessed over the telephone or through a face-to-face interview with the SIPS/SOPS.

Our clinicians referred subjects in the FE-Sz group after they were diagnosed with Sz according to the DSM-IV criteria. Subjects in the CH-Sz group were recruited from inpatient units in a psychiatric hospital. Patients were also assessed using the Positive and Negative Syndrome Scale (PANSS) [33] within the same day of being assessed using by the RBANS. All demographic and clinical information were documented from patients’ medical records. Four senior raters (a minimum of three years of psychiatric practice experience) were involved in the SIPS/SOPS, PANSS, and RBANS assessments. These 4 raters attended a 7-day training session organized by a corresponding author before the study began. All tests followed standardized testing procedures in a fixed order. Inter-rater reliability (ICC) for P symptoms from the SIPS/SOPS ranged from. 86 (P5) to. 98 (P4); the correlation coefficient between raters for the PANSS was greater than. 80.

### Data analysis

We used SPSS version 16.0 (SPSS, Inc., Chicago, IL, USA) statistical software for data analysis. Analyses of variance (ANOVAs) were used to compare PANSS scores between the FE-Sz and CH-Sz group. When significance was observed with an ANOVA on RBANS scores, the effect of age and education was corrected and Bonferroni adjustments were used for all post hoc multiple-group comparisons. To construct a predictive model of conversion risk, forward stepwise logistic regression was used on the combined samples of the CHR and HC subjects, taking into account conversion (fully psychosis) as the dependent variable and the RBANS index domains and demographic features as independent variables. We included explanatory variables with an α of less than. 10 in the univariate analyses. Pearson’s correlation coefficients were used to explore the relationship between RBANS scores and the course of Sz (the data of Sz course derived from FE-Sz and CH-Sz patients, defined as years between psychosis onset and baseline assessment in this study). We also calculated partial correlations between relevant variables by controlling for age and education. Statistical significance was *p* <. 05.

## Results

### Demographics and clinical characteristics

Age, gender, education, and marital status were not significantly different between controls and the CHR group. The majority of FE-Sz (76.9%) and Ch-Sz subjects (87.8%) were male, and the Ch-Sz subjects were much older compared with the other groups. Mean scores on the SOPS for the CHR group and PANSS measures for the FE-Sz and Ch-Sz groups are listed in Table 1. The mean time it took the CHR subjects to look for professional help once the sub-clinical psychotic symptoms began was approximately 3.8 ± 3.7 months. As for the Ch-Sz group (mean course = 28.3 years), antipsychotic drug treatment was mainly oral mono-therapy (79.6%), and clozapine was most commonly used, followed by chlorpromazine and risperidone. The mean daily antipsychotic dose, which was converted to chlorpromazine equivalents [34], was 288.7 mg. Compared with the Ch-Sz group, subjects in the FE-Sz group had significantly higher positive and general psychopathology PANSS subscale scores (*p* <. 001).

**Table 1:** Demographic and clinical characteristics.

Variables	Controls	CHR	FE-Sz	Ch-Sz
Cases (*n*)	28	27	26	147
Age (in years), [*Mean (SD)*]	26.5 (8.24)	25.04 (7.83)	23.04 (6.89)	52.5 (10.38)
Male [*n (%)*]	15 (53.6%)	15 (55.6%)	20 (76.9%)	129 (87.8%)
Education (in years), [*Mean (SD)*]	13.5 (3.31)	12.6 (3.42)	11.5 (2.61)	10.0 (2.10)
Single/separated/divorced, [*n (%)*]	16 (57.1%)	24 (88.9%)	20 (76.9%)	130 (88.4%)
Course (in years), [*Mean (SD)*]	-	-	-	28.3 (9.07)
With atypical antipsychotic type [*n (%)*]	-	-	-	126 (85.7%)
1^st^ commonly used (Clozapine) [*n (%)*]	-	-	-	66 (44.9%)
2^nd^ commonly used (Chlorpromazine) [*n (%)*]	-	-	-	32 (21.8%)
3^rd^ commonly used (Risperidone) [*n (%)*]	-	-	-	29 (19.7%)
Antipsychotic dose ^a^ (mg/d)	-	-	-	288.7 (178.26)
**SIPS/SOPS**				
Positive symptoms, [*Mean (SD)*]	-	8.8 (4.45)	-	-
Negative symptoms, [*Mean (SD)*]	-	10.1 (5.99)	-	-
Disorganized symptoms, [*Mean (SD)*]	-	4.2 (2.45)	-	-
General symptoms, [*Mean (SD)*]	-	8.0 (2.50)	-	-
**PANSS**				
Total score, [*Mean (SD)*]			81.0 (15.12)	58.7 (12.32)
Positive symptom subscore, [*Mean (SD)*]	-	-	21.0 (5.58)	10.2 (4.44)
Negative symptom subscore, [*Mean (SD)*]	-	-	21.3 (5.35)	21.3 (6.80)
General psychopathology subscore, [*Mean (SD)*]	-	-	38.8 (7.38)	27.2 (5.85)

*Note*:

^a^ Chlorpromazine-equivalent antipsychotics.

### Cognitive performance in the control, CHR, and FE-Sz patient groups

The mean of the RBANS domain index scores for controls, CHR, and FE-Sz patients are shown in Table 2. Overall, the RBANS total score and five index scores were significantly different among these groups. The FE-Sz patients exhibited more severe dysfunction in memory (immediate and delayed), language, and attention relative to the CHR subjects. Although mean scores on the RBANS were lower among the CHR subjects compared to controls, differences were not significant at the. 05 level, except for the visuospatial domain.

**Table 2:** A comparison of RBANS domain index scores between controls and CHR and FE-Sz patients.

RBANS Domain	HC		CHR		FE-Sz		*F*		*p* *(HC vs. CHR vs. FE-Sz)	*p* (HC vs. CHR)	*p* (HC vs. FE-Sz)		*p*(CHR vs. FE-Sz)
**Immediate Memory**													
Mean (SD)	96.36 (13.08)	95.07 (15.20)		72.31 (16.35)		20.08		<. 001		1	<. 001	<. 001	
Median (range)	94 (76–123)	97 (53–126)		77 (40–106)		-		-		-	-	-	
**Visuospatial/Constructional**													
Mean (SD)	106.82 (10.66)	93.67 (18.25)		87.15 (17.77)		8.78		<. 001		.013	<. 001	.646	
Median (range)	105 (84–121)	92 (62–121)		92 (53–121)		-		-		-	-	-	
**Language**													
Mean (SD)	100.89 (10.04)	94.48 (12.35)		84.85 (12.66)		10.07		<. 001		.214	<. 001	.022	
Median (range)	101 (84–121)	96 (74–116)		85 (51–120)		-		-		-	-	-	
**Attention**													
Mean (SD)	106.36 (13.06)	104.89 (17.90)		91.96 (16.94)		6.49		.002		1	.005		.009
Median (range)	112 (79–128)	106 (56–132)		94 (56–122)		-		-		-	-	-	
**Delayed Memory**													
Mean (SD)	103.50 (6.51)	95.41 (11.53)		81.27 (19.19)		16.62		<. 001		.113	<. 001	.001	
Median (range)	103 (94–118)	97 (56–123)		85 (44–105)		-		-		-	-	-	
**RBANS Total Scale Index Score**													
Mean (SD)	103.32 (10.99)	95.15 (14.09)		78.69 (15.84)		20.72		<. 001		.122	<. 001	<. 001	
Median (range)	104 (85–124)	95 (55–119)		85 (46–101)		-		-		-	-	-	

* Adjustment for multiple comparisons: Bonferroni.

### Prediction of conversion based on RBANS results

As shown in Table 3, forward stepwise logistic regression for the sample of CHR and healthy controls were used to identify which of the RBANS domains were most predictive of conversion. The presence of psychosis was listed as the dependent variable while age, education, and the RBANS domains were listed as independent variables. Age and delayed memory were found to significantly predict conversion to psychosis in this model.

**Table 3:** Logistic regression for predicting the transition to psychosis.

Predictor Variable	Beta	S.E.	Odds Ratio	95％CI	Wald statistic	P value
**Age**	.792	.366	2.208	1.077–4.526	4.677	.031
**Delayed Memory**	.358	.171	1.430	1.022–2.000	4.354	.037

### Cognitive decline at different stages during the course of psychosis

Relationships between the RBANS domain index scores and the course of Sz are presented in Fig 2. The Ch-Sz group were divided into middle-term (≤ 27 years, 27 years is the median) and long-term (> 27 years) groups according to the course of Sz. Overall, the RBANS domain scores declined along with disease course, but rates of decline were not consistent. The immediate memory domain seemed to have declined more robustly after the onset of psychosis, but the visuospatial domain seems to decline more rapidly during the prodromal stage. The decline trends for the delayed memory domain and total index scores seem to be similar and synchronized.

**Fig 2:** RBANS results at different stages during the course of psychosis. The RBANS domain index scores (y axis) is plotted against the course of Sz (x axis). RBANS scores declined along with disease progression. The trajectory of delayed memory decline is consistent with RBANS total scale index score.

### The course of Sz related to cognitive performance

To determine if the course of Sz, age, and education was associated with cognitive abilities, correlations between the RBANS total and index scores and the course of Sz are shown in Table 4. These correlations demonstrate that the RBANS indices were highly associated with disease course, age, and education. However, after controlling for age and education, partial correlations showed that the only significant link was between delayed memory and the course of Sz.

**Table 4:** Correlations between the course of Sz and RBANS domain index scores.

	Immediate Memory	Visuospatial/ Constructional	Language	Attention	Delayed Memory	RBANS Total Scale Index Score
Course	-.28	-.19	-.10	-.28	-.25	-.29
*p* (*df* = 171)	<. 001	.011	.184	<. 001	.001	<. 001
Age	-.23	-.16	-.06	-.22	-.16	-.22
*p* (*df* = 171)	.002	.039	.404	.004	.035	.004
Education	.283	.279	.123	.295	.247	.329
*p* (*df* = 171)	<. 001	<. 001	.106	<. 001	.001	<. 001
Controlled for Age & Education (partial correlation)						
Course	-.10	-.04	-.06	-.12	-.16	-.13
*p* (*df* = 169)	.197	.574	.436	.105	**.032**	.095

## Discussion

The current study assessed neuropsychological performance, as measured by the RBANS, among several patient groups in various stages of psychosis. To our knowledge, no previous study has reported on the cognitive profiles of psychotic patients from the prodrome stage to long-term chronic psychosis. In line with our hypothesis, the current study further supported that cognitive impairment among patients with psychosis is broad, and increasingly severe cognitive deficits emerge the longer the disease progresses. More importantly, and contrary to other neuropsychological functional domains, delayed memory was statistically related to the development of psychosis during both pre-onset and post-onset stages.

Compared with the FE-Sz and HC groups, our data showed that deficits in neuropsychological performance identified in the CHR samples characterized by a modest level of severity that is intermediate between HC individuals and FE-Sz patients, especially when comparing with the FE-Sz group where more severe cognitive impairment emerged. Although differences between the CHR and HC groups were not significant (except for the VC domain), trends in decline (and group differences) were observed, which implied that cognitive deficits might already be present prior to the onset of full psychosis. Consistent with several recent longitudinal studies [15, 35, 36], cognitive performance among the Sz patients was worse when compared to the CHR subjects. Based on the baseline assessment and 2-year follow-up with the CHR subjects, younger patients with poorer delayed memory might be expected to progress toward full psychosis within 2 years. Only a few studies to date have assessed cognitive function among CHR groups [15, 37, 38] and have examined the value of predicting later psychosis. For instance, failures in olfactory identification [39], memory [40–42], and language function [43] domains have been predictive of the future onset of full psychosis. Partly consistent with such findings [40], we found that only delayed memory deficits could be somewhat predictive in identifying those at high risk for a Sz spectrum disorder. Considering these findings with a disease etiology point of view, memory functioning impairment might increase vulnerability to environmental influences and impact insights related to psychotic experiences [6].

It must be noted that cognitive impairment is not a specific symptom and is broadly present at every stage of psychosis. Therefore, investigating declines in cognition from a comprehensive sample covering different courses of psychosis is likely more useful for understanding the progression of cognitive dysfunction. Our findings revealed that those individuals with longer Sz disease courses had poorer neuropsychological performances. This was not unexpected and highly consistent with other studies [5, 36, 44]. Surprisingly, only delayed memory was significantly related to disease course and general cognitive ability (total RBANS score). If reliable, these findings would imply that delayed memory might reflect an important endophenotype of psychosis onset, as well as disease progression, which manifests in early neurodevelopmental impairment. Toulopoulou [45] reported a link between delayed verbal memory and left hippocampal volume among patients with Sz, hence confirming that cognitive deficits might be overlaid to the underlying neuropathological development observed in psychosis.

Delayed memory decline has been observed in several studies [46–48] of patients with Sz as well as prodromal subjects [40]. Other studies [7, 49] have also found that memory functioning is positively related to social role functions. Our results further support previous findings showing that delayed memory ability might be more specifically impaired during all psychotic phases. Clinically, interpreting our results in the context of previous findings, it may be worthwhile for clinicians to chart each participants’ memory functioning [14], from the prodromal stage to later stages of psychosis. Clinicians should be aware that subjects with psychotic experiences may require specific monitoring or support in their memory functions related to psychosis emergence and progression. Since the trajectory of delayed memory decline is consistent, which also reflects the development of psychotic illness, charting individual memory functioning over time from the prodromal stage to later stages is necessary and beneficial.

Although we included psychotic patients through all stages to obtain a more refined picture of cognitive decline, this study does have some limitations. First, our subjects were screened and interviewed by clinical diagnostic instruments such as the SIPS/SOPS, PANSS, etc. However, no objective intelligence quotient (IQ) test was applied during the screening procedure. Whether this limitation affects the present findings regarding discrepancies in cognitive deficits is unknown. Second, the majority of our sample in the Fe-Sz and Ch-Sz groups was male. Beatty and colleagues [50] reported gender differences on the RBANS test in a community sample. They found non-clinical females perform better than males on measures of memory functioning. Thus, whether our results regarding post-onset phases of Sz also apply to female patients with Sz warrants further investigation. Third, the relevancy of using antipsychotic medicine in the Ch-Sz cohorts is still an indecisive answer; however, several studies [51, 52] provide supporting evidence related to this issue. Fourth, chronic patients with Sz in this study were from inpatient units in a psychiatric hospital, it is not known if these findings can be generalized to primary care or outpatient settings.

Despite these limitations, our study explored cognitive changes through all phases of psychosis whereby cognitive deficits were broadly observed and followed by the progression of psychotic diseases. Impairment in delayed memory was the most common deficit and was the most sensitive to disease progression. Future studies should examine the potential effectiveness and feasibility of implementing cognitive enhancement training and monitoring for psychotic patients in clinical settings.
